RETRACTED

# Detection of Types of Mental Illness through the Social Network Using Ensembled Deep Learning Model

**DOI:** 10.1155/2022/9404242

**Published:** 2022-03-26

**Authors:** Syed Nasrullah, Asadullah Jalali

**Affiliations:** ^1^Department of Information Systems, College of Computer Engineering & Sciences, Prince Sattam Bin Abdulaziz University, Al-Kharj 11942, Saudi Arabia; ^2^American University of Afghanistan, STM (Science Technology Mathematics), Kabul, Afghanistan

## Abstract

In today's era, social networking platforms are widely used to share emotions. These types of emotions are often analyzed to predict the user's behavior. In this paper, these types of sentiments are classified to predict the mental illness of the user using the ensembled deep learning model. The Reddit social networking platform is used for the analysis, and the ensembling deep learning model is implemented through convolutional neural network and the recurrent neural network. In this work, multiclass classification is performed for predicting mental illness such as anxiety vs. nonanxiety, bipolar vs. nonbipolar, dementia vs. nondementia, and psychotic vs. nonpsychotic. The performance parameters used for evaluating the models are accuracy, precision, recall, and F1 score. The proposed ensemble model used for performing the multiclass classification has performed better than the other models, with an accuracy greater than 92% in predicting the class.

## 1. Introduction

Many people use social media to express their emotions and thoughts [1]. Users frequently share their mental health difficulties or illnesses anonymously on numerous social media platforms or online social health forums [2]. It is possible to express sympathy for individuals with comparable symptoms by joining an online health community. Users also frequently utilize social media to gather information about their symptoms in an attempt at self-diagnosis. Numerous academics have used social media to study people's emotional states and mental illnesses, including depression, anxiety, and schizophrenia. According to the study, recent research gathered tweets from people who had reportedly been diagnosed with depression. Linguistic Inquiry and Word Count (LIWC) was a tool used to analyze and track changes in social interaction on Twitter using the collected messages [3]. To better understand the risk of postpartum depression among Facebook users, another study used specialized psychometric measures to compare the levels of postpartum depression between the pre-and postnatal periods. Reece et al. [4] analyzed image data to predict social network users' depression in their research. Instagram images were analyzed with face identification and colorimetric analysis. Exploring user posts and N-gram language modeling and vector embedding techniques helped a prior study predict who might develop anxiety illnesses in the future [5].

RETRACTED

Several prior research found that social media data efficiently monitored or detected users' moods or prospective mental health issues. This study's objective is to build a deep learning model that can detect various mental health problems in users by accumulating social media-related mental health-related data such as depression, anxiety, BPD, schizophrenia, and autism. Groups (or “subreddits”) such as r/depression and r/bipolar were employed to acquire data from Reddit users. We collected data from six subreddits that deal with mental health issues, including bipolar, psychiatric disorders (such as schizophrenia and bipolar disorder), and autism, to determine if someone is depressed or anxious [6]. The subreddits that have been previously researched were utilized in this analysis. Mental health-related subreddits were discovered among the most popular subreddits using a statistical methodology such as a semisupervised method and an assessment procedure by experts. Subreddits such as R/depression and all others related to depression are examples of this.

Reddit's mental health subreddits helped us determine if individual posts could be classified as relevant forms of mental illness. The symptoms of depression and bipolar disease are so similar that patients with particular mental disorders may not recognize their most appropriate diagnosis due to the difficulty in diagnosing bipolar disorder. At first glance, we felt that people were seeking help by opening up generic stories about themselves by using phrases such as “mental health,” “mental ailment,” or “mental state.” Initially, individuals are more likely to communicate with others on Reddit in a general health-related channel, but they fail to recognize the unique health issues discussed there. Consequently, we are trying to identify social media users who may be suffering from mental health problems [7]. This investigation aims to answer the following research question.

According to the World Health Organization (WHO) Mental Disorders Fact Sheet in January 2020, more than 264 million individuals of all ages suffer from depression [8]. COVID-19's spread has also been connected to increased mental health disorders. It's only a matter of time before more people get the treatment they need for depression. Suicide is a leading cause of death among people aged 15 to 29 due to a shortage of resources for those who have a mental illness. Every year, more than 80,000 individuals die due to this dearth of medical care. There has been a steady rise in major depressive episodes among adolescents in the United States over the past decade. Mental illness is predicted to have a global economic impact of more than 5 trillion dollars by the year 2030, according to projections [9]. It's quite evident that preventative and intervention approaches are in demand.

RETRACTED

Researchers have found that a growing number of people are using social media sites such as Twitter and Facebook to express themselves and connect with others in real-time [10]. As a result, a massive amount of social data is generated, containing traces of useful information about people's preferences, moods, and activities. About 57 percent of the world's population is predicted to be using social media by the year 2021, according to Hootsuite. Over the past year, the number of unique users worldwide has increased by 520 million, or more than 13 percent on an annual basis. According to Conway and colleagues, people's health monitoring and mental health applications have used social media data as a data source. Because of their usefulness as medical decision support systems and the difficulty of diagnosing mental disorders using traditional approaches that rely primarily on surveys and interviews, online screening tools that can analyze indications of mental disorders are valuable. As a result, new screening tools for mental disease can be developed by predicting well-known symptoms from social media data. Several studies have proven, for example, that language patterns can serve as an indicator of a person's mental health state utilizing machine learning techniques.

The following is a general outline of how deep learning techniques are used in research: There are three steps involved in this process: creating a file of various types of mental illness diseases, fitting a model based on that data, and testing estimation accuracy concerning that data. An absence has hindered research on applied mental health issues in the number of datasets available. Crisis informatics, rapid diagnosis, action, and effective treatment can benefit from a solution to this problem. Because recognizing risk factors for mental illness often necessitates quick action, creating successful intervention programs is hampered by these gaps in time. Mentally ill individuals may also have less cooperation with the research team. Textual elements (especially tweets) dominate the reviews, but many other types of social data can investigate psychological signals [11]. For example, visual qualities have received relatively little attention. According to certain studies, photographs are the most popular content posted on social media platforms, despite their enormous volume. Many concerns remain unresolved concerning the social data on mental illness, a relatively new field of study.

RETRACTED

The paper's organization is as follows: Section 1 describes the introduction, and section 2 covers the literature survey. Then, in section 3, proposed methodology is explained, and section 4 shows the result. Finally, the last section describes the conclusion and future work, followed by the reference section.

## 2. Literature Survey

Data collection methods in the field of social media-based mental illness prediction can be divided into two categories: (1) collecting data directly from users with their permission, using surveys and data collection tools, or (2) extracting data from public posts through APIs (application programming interfaces). First, researchers used crowdsourcing platforms or data donation websites such as OurDataHelps to post research information and invite users to participate in the application by filling out questionnaires and consenting to collect their social data. Two of the most commonly used questionnaires for measuring depression are the Center for Epidemiologic Studies Depression Scale (CESD) and the Beck Depression Inventory (BDI). To detect suicidal ideation, the Suicide Probability Scale (SPS) and the Satisfaction with Life Scale (SWLS) can be useful instruments [12]. Since social media platforms' APIs allow developers to access public data, the second approach collects related posts by using keywords or regular expressions associated with those keywords or phrases. Self-reported diagnosis can be defined as the use of regular expressions such as “I was diagnosed with (disorder)” for a variety of mental health issues in the postretrieval process. APIs lead to a collection of posts that need to be analyzed before they can be used in further research. Suicide ideation denial, discussion of other people's suicide, or news or reports about suicide are considered irrelevant and removed from the collection if they contain relevant keywords/phrases. Only posts containing hypothetical statements, rebuttals, or quotations are considered positive samples in the self-report diagnosis process.

A common approach to validating regular expressions is with human annotators, which many researchers suggest, given the issues we discussed in the introduction. Predefined datasets, such as those from the myPersonality project, the Computational Linguistics and Clinical Psychology (CLPsych) [13], and the eRisk workshops [14], can also be used to collect data, as can other methods of collecting test scores and social data. Before the actual analysis, most studies preprocessed the collected data by removing stop words, tweets, hashtags, and URLs as well as lowercase characters [15]. ASCII-converted emojis were also used to facilitate future analysis of the data. Selecting only the most relevant features after feature extraction reduces training time, stimulates interpretation, and increases the likelihood that the model will generalise and avoid overfitting [16]. Support vector machines (SVMs) and a variety of kernels, such as linear and radial basis functions (RBFs), as well as different types of regression, such as linear, log-linear, and logistic, as well as nave Bayes, decision trees, and random forests, are the most widely used machine learning methods for predicting mental disorders [17]. People with depression and suicide-related psychiatric stressors have also been studied using deep learning approaches [18]. Even though feature normalisation and parameter tuning were not well documented in most previous studies, the evaluation mechanism is used to assess the classification model's reliability after prediction. Several metrics and visualisation tools in the literature can be used to evaluate the performance of proposed models, such as classification accuracy, confusion matrix, precision, recall, F1 score, and receiver operating characteristics curve (ROC).

RETRACTED

According to a few studies, machine learning methods can identify relevant features [19]. The study of new features that can be used to train a classifier and lead to discovering hidden patterns and relationships in the data is the primary focus of this research, not the development of learning methods. When it comes to mental illness, most research relies on textual content and linguistic patterns. NLP methods, such as those developed by Coppersmith et al. [20], can gain insights into specific mental health disorders, such as PTSD; depression; bipolar disorder; and seasonal affective disorder (SAD). They also emphasised the strong connection between mental disorders and language patterns, such as first-person pronouns, anger words, and other negative emotions. Linguistic Inquiry and Word Count (LIWC) analysis contributed to these findings. With the help of dictionaries that cover various psychological categories, it has been manually built by psychologists. For instance, this technique could extract personal pronouns and positive/negative emotions from the text. Also, popular sentiment analysis tools, SentiStrength [21] and OpinionFinder [22], were used in selected research papers to measure the sentiment of textual expressions [23]. Latent Dirichlet Allocation (LDA) is a topic modeling technique that has been used in several efforts to uncover latent topics from user postings [24].

RETRACTED

Despite this, most studies focus on textual features, with only a few incorporating image analysis techniques. For example, Kang et al. used colour compositions and SIFT descriptors as visual features to extract emotional meanings from a Twitter image [25]. Using the image's hue, saturation, and brightness, Reece et al. [4] can predict Instagram users' signs of depression. As Guntuku et al. [26] have shown, using the VGG-Net [27] image classifier can also be used to predict depression in more recent studies.

In the above discussed paper, the focus was on multiple convolution neural network and these networks takes much amount of time during the analysis. So, this proposed work has used the limited number of convolution neural network for the extraction of the features and later on recurrent neural network is used for performing the classification.

## 3. Proposed Methodology

In this work, 4 different types of classification have been performed based on the mental illness. The four diseases taken for the classification are anxiety_vs_non_anxiety, bipolar_vs_non_bipolar, dementia_vs_nondementia, and the psychotic_vs_non_psychotic. These four diseases are classified using the deep learning model based on the Ensemble deep learning models. The novelty of this work is to apply the ensembled approach using the LSTM model and the convolutional neural network for performing the classification of different types of mental illness. Let us discuss the proposed methodology in detail.

### 3.1. Dataset

The dataset has been collected from the reddit using NLTK python library. The dataset consists of 301746 records with labels such as anxiety_vs_non_anxiety, bipolar_vs_non_bipolar, depression_vs_non_depression, and the psychotic_vs_non_psychotic. The dataset will be processed through different process such as data cleaning and lemmatization. The most common category of mental health disorders in America impacts approximately 40 million adults 18 and older. Most parts of the dataset are taken from the research paper [6].

### 3.2. Ensemble Deep Learning Models

In this work, two recurrent (bidirectional LSTM) and one convolutional neural network is used for performing the classification. In the first stage, dataset is preprocessed and then, the preprocessed data are passed through multiple deep learning models such as recurrent neural network and convolutional neural network.  Figure 1 shows the flowchart of the proposed work, and the proposed methodology is discussed in detail.

#### 3.2.1. Word Embedding through Continuous Bag of Words Model (CBOW)

In natural language processing, Word2vec is widely regarded as a breakthrough. As a result, it is widely accepted and widely used. An embedding technique called Word2vec is utilized to turn the dataset's text into vector form, which a computer can recognize. There is a vector for every word in your dataset, and the size of the vectors varies with word length. For the CBOW model, context is considered and used as an input. Afterwards, it tries to forecast words that are relevant to the context. When it comes to this, let us look at an example. In this example, the neural network receives the word “depression” as an input and processes the sentence, “Help with rejection, depression, suicide issues.” Predicting the word “depression” is what we are aiming for with this exercise. Input words will be encoded with one-hot encoding, and the error rates of the encoded target word will be measured. Predicting the result based on the term with the least error is easier if we do this.

RETRACTED

The above diagram depicts the CBOW model's architecture. Understanding the context of surrounding words helps the model anticipate a target word. This line, “Help with rejection, depression, suicide issues,” is a good example. This sentence is broken down into word pairs using the approach (context word, target word). The user must customise the window size. For example, if the context word has a 2-word window, the word pairings would be as follows: ([help, with], rejection), ([with, rejection], depression), and ([rejection depression], suicide). When making predictions with this set of word pairs, contextual terms are taken into account. The input layer will consist of four 1XW input vectors if we employ four context words to predict a single-target word. A WXN matrix is used to multiply these input vectors in the buried layer. An element-by-element summation of the 1XN hidden layer output to produce the final activation and output, as shown in Figure 2.

#### 3.2.2. Convolutional Neural Network

In this work, a single CNN model is used for performing the analysis. The input training samples are fed into convolution layers, which extract features. Each convolution layer has a set of filters that aid in extracting features. In general, the complexity of features learned by convolution layers increases as the depth of the CNN model increases. For example, the first convolution layer focuses on simple features, while the last layer focuses on more complex features of training samples. When extracting features, the convolution of a portion of the data sample is considered. Stride length and padding value determine how much data the filter can process at a given time. Before convolution, data samples may or may not be subjected to zero padding. An activation unit called ReLU is used further to process the convolutional output (rectified linear unit). The data is transformed into a nonlinear form by this unit. The ReLU output is clipped to zero when the convolution output is negative. The vanishing gradient problem prevents sigmoid units from being used as activation units. If the depth of CNN is large, the gradient found at the input layer will have diminished greatly when it reaches the output layer. As a result, the network's overall output varies slightly. As a result, the convergence rate is either slow or nonexistent. ReLU is preferred to avoid such a situation.

RETRACTED

After that, a pooling layer receives the ReLU's output. During convolution, a pooling layer removes any redundant features that were captured. As a result, the data sample is smaller thanks to this layer. Pooling is based on the assumption that the values of adjacent pixels in an image are nearly identical. Pooling is performed using the average, minimum, and maximum four adjacent pixel values. Using a 2*∗*2 filter, the size of the input image is reduced by half. Before pooling, the input data may or may not be subject to zero padding. In the CNN model, this convolution and pooling layer is repeated. Also, it is repeated 2–4 times for educational purposes. Multilayer neural networks are used to process the output of the convolution and pooling layers. In this case, each neuron unit serves as a feature map for a particular unit. By making the CNN model noise-resistant, the dropout layer reduces overfitting. Layers like these are typically inserted between two layers of a neural network that are already fully connected. As a result, they temporarily disrupted data flow between two completely interconnected systems. This is the same as teaching the model to classify under noisy conditions accurately. As a result, the likelihood of an overfitted model classifying incorrectly decreases. The SoftMax function is used to compute the CNN model's output. Rather than just ≥ 0.5 for sigmoid output, SoftMax provides the probability of outputs for various classes. The use of SoftMax to find output results based on the most likely class increases output accuracy. The model is mathematically discussed as follows.

Using *L* and *V* as sentence and word vector lengths measures is common. Let *S* ∈ *R*^*L*,*V*^ be the sentence matrix. It is necessary to apply a convolutional kernel *C*  ∈  *R*^*L*,*W*^ to an array of *W* words before the new feature can be produced using a convolutional operation. There are many ways to generate features such as *F*_*i*_, from S [*∗*, *i* : *i*+*W*] such as

(1) $$\begin{array}{c} F_{i}=\sigma \left(\sum^{}\left(\text{S}\left[*,i:i+W\right]ο\;C\right)+b\right). \end{array}$$

In the above equation (1), *σ* is the nonlinear function and *b*  ∈  *R* is a bias term. In this work, ReLu is the nonlinear function and *ο* is used to represent the Hadamard product. Hadamard product of two matrices is “To generate a feature map, the convolutional kernel is run on every possible combination of words in the sentence. To identify the most important feature in the feature map, we perform a pairwise max-pooling operation. The pooling operation can be viewed as feature selection in natural language processing. A max-pooling operation is also performed and specifically the feature map, which results from convolution *F*=[*F*_1_, *F*_2_,…, *F*_*L*−*W*+1_] is the pooling operation's input. Allowing for a two-fold reduction in input, let's calculate these two adjacent features in the feature map as follows:

(2) $$\begin{array}{c} M_{i}=\max\left(F_{2xi-1},F_{2xi}\right). \end{array}$$

Maximizing the pooling operation yields the following output:

(3) $$\begin{array}{c} M=\left[M_{1},M_{2},\ldots \ldots \ldots .M\frac{L-W+1}{2}\right], \end{array}$$

where *M* ∈ *R*^(*L* − *W*+1/2)^.

RETRACTED

#### 3.2.3. Recurrent Neural Network

For the most part, our classification model is based on an attention-based Bi-LSTM architecture. Each word has a unique correlation with final classification, even though CNNs reduce input features to be used for prediction. We plan to use CNN and Bi-LSTM to their full potential in this study. As a result, the Bi-LSTM is able to encode word dependencies over long distances more effectively.  Figure 1 depicts the Bi-LSTM process. Using the CNN stage's features, it extracts the final hidden layer to generate new features. The information obtained by Bi-LSTM can be viewed as two different textual representations because it has access to both the preceding and subsequent contextual information. A Bi-LSTM model generates a representation of the sequence using the features obtained from the CNN. In the end, the attention layer selects the most correlated features to use for final classification. For “I'm angry. I'm angry at myself,” the attention mechanism assigns more weight to “angry” and less weight to “myself” in order to classify the sentence as depression. The point is to demonstrate that despite the illness's negative impact, the “angry” attitude remains unfazed. The attention mechanism improves prediction accuracy and reduces the number of learnable weights required by this process. This model's attention mechanism uses the Bahdanau attention with the following:

(4) $$\begin{array}{c} \text{score}\left(\text{query},\text{key}\right)=\;V^{T}\text{tanh}\left(W_{1\text{key}}+W_{2\text{key}}\right). \end{array}$$

RETRACTED

## 4. Results and Discussion

The proposed work is implemented through Python programming language. The parameters used for the evaluation of the performance of the models are accuracy, precision, recall, and F1 score.

Table 1 has shown the comparison of the existing model with the proposed ensembled model. The table has shown that the proposed model has performed better than the existing model based on convolutional neural network.

Figure 3 has shown the accuracy comparison of the proposed work. Using this work, bipolar mental illness can be classified more accurately than other types of mental illness.

## 5. Conclusion and Future Work

In this paper, different types of mental illness are classified using the deep learning model. The ensemble deep learning model is implemented using convolutional neural network and the recurrent neural network for organizing mental illnesses such as anxiety, bipolar, dementia, and psychotic. The ensemble deep learning model has performed better than the existing models, based on the parameters such as accuracy, precision, recall, and F1 score. In future work, different types of convolutional networks such as capsule network can be implemented to classify mental illness using images.

## Figures and Tables

**Figure 1:** Flowchart of the proposed work.

**Figure 2:** Architecture of CBOW word embedding model.

**Figure 3:** Accuracy comparison of the proposed work.

**Table 1:** Comparison table of the deep learning models.

Channel	Class	CNN				Ensemble deep learning model			
		Accuracy (%)	Precision	Recall	F1 score	Accuracy	Precision	Recall	F1 score
Anxiety	Anxiety	77.81	87.54	41.44	56.25	80.13	89.63	50.14	64.30
	Nonanxiety		75.92	96.91	85.14		77.16	98.13	86.39
Bipolar	Bipolar	90.20	87.22	38.02	52.95	92.14	89.13	45.42	60.17
	Nonbipolar		90.40	99.05	94.53		92.56	99.43	95.99
Dementia	Dementia	75.13	89.1	71.75	79.49	80.45	90.46	76.17	82.7
	Nondementia		58.66	82.04	68.41		64.23	86.04	73.55
Psychotic	Psychotic					78.85	83.45	61.23	70.63
	Nonpsychotic						76.73	70.94	73.75

## Data Availability

The dataset has been collected from the reddit using NLTK python library.
